# Quality supervision mechanisms on green product for online retailing in the blockchain technology era

**DOI:** 10.1371/journal.pone.0306093

**Published:** 2024-07-24

**Authors:** Hong Wang, Yuheng Xu

**Affiliations:** School of Economics and Management, Nanjing Forestry University, Nanjing, Jiangsu, China; Beihang University, CHINA

## Abstract

With the development of e-commerce and the increase of consumers’ green consciousness, more and more consumers purchase green products online. The frequent occurrence of the fake green product in online shopping has been harmful to the management and operation of the online market. In order to find the ways for the platform to supervise effectively green products quality problems, we consider the role of blockchain technology, the dynamic penalty mechanisms, the three strategy choices of seller, and the green awareness of consumers, and establish a supervision game model with the participation of online platform, online seller and consumer, which analyzes the equilibrium state of the three parties. The results show that (1) the level of the consumers’ green awareness, the compensation for green consumers, and the cost saved by non-green products are the critical factors to ensure the effectiveness of the platform punishment mechanism; (2) the combine effect of dynamic punishment and blockchain supervision can effectively and rapidly improve the quality of green products; (3) the improvement of consumers’ green awareness can drive sellers to sell green product, and makes the platform to strengthen the supervision of fake green products.

## 1. Introduction

Recently, with the improvement of the consumers’ green awareness, online green product quality problems have been concerned by consumers. The China Sustainable Consumption Research Program in 2023 shows that 83.4% of Chinese consumers have realized the importance of green consumption. More than 60% of consumers choose to purchase green products on online platform. Green consumption is imperceptibly influencing consumers’ purchase behavior. E-commerce platform becomes the most popular green consumption channel. However, due to the limitation of traditional inspection supervision, it is impossible for platform to inspect all green products. By comparison with physical stores, online platforms can offer a low price and a convenient shopping experience. However, consumers are more difficult to identify the product’s actual quality. This means that sellers can easily manipulate the information about green product quality. It can be an easy job to disguise fake green products as green products. The government has taken some measures and actions to supervise online green product. However, due to the high cost and low efficiency, the government is difficulty to establish a suitable mechanism to oversee online product quality. In contrast with the government, the online platform has more advantages in collecting and processing transaction data. But most of platforms cannot adopt more suitable penalty mechanisms, it also contributes to the lower penalties of selling fake green products.

According to the E-commerce Law of the People’s Republic of China, online platform has more responsibility to supervise the product quality and protect consumers’ rights. In reality, numerous online platforms (e.g., JD.com and Amazon) have taken measures to mitigate information asymmetries, such as online green product reviews and labeling [1]. Even though online platforms can provide more information about product quality, consumers still bear product quality uncertainty risks. Fortunately, Blockchain technology can better solve the information asymmetry issues because of its integrity, transparency, and security of information [2]. It has been applied to the luxury supply chain [3], the food supply chain [4] and fresh product supply chain [5]. Wal Mart applied blockchain technology to fresh food, private brands and other categories, and took the lead in building a pork and beef traceability platform project. The platforms also like Alibaba and JD.com in China have announced to ensure authenticity for some products by blockchain technology [6], and heavy penalties imposed on the bad behaviors of sellers, such as JD punishes counterfeits with a penalty. The purpose of this study is to answer the following questions:

1. Which quality supervision mechanisms dominated by the online platform can effectively solve the green product quality problems?
2. What are the key factors that affect the platform’s adoption of punishment mechanisms?
3. What role can consumers’ green awareness play in platforms’ supervision and the production of sellers?

In view of this, this paper considers the role of blockchain technology, the dynamic penalty mechanisms, three strategy choices of seller, and the green awareness of consumers, establishes a supervision game model to explore an effective way to regulate the green product quality issues on the platform.

This paper can be organized as follows: Section 2 reviews the relevant literature. Section 3 introduces the basic assumptions, and analyses the evolutionary strategies of three players. Section 4 simulates and discusses the effects of different penalty mechanisms. Section 5 concludes this paper, and advices future research.

## 2. Literature review

Our work is most closely relevant to the research on quality information disclosure and quality supervision.

### 2.1 Quality information disclosure

Quality information disclosure has been studied by pieces of literature. A few factors are examined in their influence on players’ disclosure strategy, such as disclosure cost [7, 8], consumers’ preference [9, 10], and competitive market [6, 11].

Some studies about quality information disclosure focus on costly quality disclosure and competitive markets. Liu et al. found that more accurate information available can push sellers to increase the retail prices, which shows the downsides of information available for consumers [12]. Markopoulos and Hosanagar considered endogenous quality production, costly quality disclosure, and information availability by third parties, the results showed that information by third parties is conducive to reducing quality disclosure investment, which favors low-quality more than high-quality firms [13]. Tan Y et al. considered competitive market structures and consumer preferences, they found that when the market is filled with heterogeneous consumers and cost of disclosure is low, competition actually hinders sellers from engaging in quality disclosure [8].

A few studies also pay attention to the impact of consumer preferences on quality information disclosure. They considered the uncertainty of consumer preferences [14]. For example, Consumers are willing to pay a premium for more product information about the qualification, credibility, and capability of sellers [15]. Zhang and Li incorporated consumer loss aversion into firms’ quality disclosure decisions. They found that as consumers become more averse to loss, symmetric firms should invest more in quality disclosure to alleviate consumer uncertainty and loss aversion [16].

The quality of product information disclosure is primarily determined by the seller. Suppliers always prefer mandatory disclosure, while the retailers’ preference depends on the price and the demand [17], which indicates that market information is asymmetric, and the essence of quality supervision is to reduce uncertainty through supervision mechanisms [18]. A few studies recently discussed the effect of blockchain to realize information disclosure [2, 19]. Considering the use of blockchain technology in e-commerce platforms, Song et al. divided the sellers’ decisions into four scenarios and established a game model to analyze the influence of blockchain technology on product information disclosure of merchants on online platforms [20].

### 2.2 Quality supervision

Product quality supervision is not only a hot topic in academic research, but also a problem that needs to be solved urgently in practice. The government plays a significant role in quality supervision, including food safety, drug quality, health product quality, and agricultural product quality. Compared with the production cost of brown product, the introduction of green product requires a launching investment [16]; green product does have moral advantages while it has disadvantages in price [21]. Consumers’ high environmental awareness will induce enterprises to produce new green products [22], but now only 27.6% of consumers can match the purchase intention to behavior [23]. They show the necessity of government regulation. For example, Sun et al. established a game model about public goods among suppliers, consumers, and the government to analyze the impact of government incentives to the suppliers’ supply and consumers’ purchase [24]. Strict enforcement of regulations by the government is an effective incentive measure [25–27]. Zhang and Georgescu established an evolutionary game theory model of farmers, their customers, and the government to control the organic food quality. They found that the government should provide strong support for organic farmers [28]. Other scholars have also taken the introduction of the mass media [29], third-party agencies [30], consumer feedback [31, 32], as well as rewards and penalties into account to solve quality issues.

Evolutionary game theory is commonly used to the supervision issues [33, 34]. He and Zhu built a three-parties evolutionary game model and discussed a consumer feedback mechanism in green product online shopping [35]. For online agricultural products quality issues, consumer evaluation and complaint feedback were introduced to an evolutionary game model about green product quality supervision with the participation of the governmental supervision department, e-commerce platform, online seller, and consumer [33]. Yang, Xie and Ma established a tripartite game model of the producers, sales operating enterprises, and local governments to analyze the behavior of the parties and the influence of brand construction to rural revitalization [36].

The theoretical contributions of this study are mainly reflected in the following aspects.

First, prior studies only consider whether the consumers purchase or not. The reality is that the growing number of environmentally conscious consumers provides significant opportunities for green product development [37], we consider the degree of consumers’ green awareness. Meanwhile, blockchain has been widely applied in many areas [38], and we consider the effect of blockchain technology into the online green product quality supervision.

Second, most of existing studies only consider green products and non-green products. They also neglected the reality that sellers sell fake green products in pursuit of profits. This paper considers the situation of the fake green products supplied by sellers.

Third, most of the penalty parameters are fixed in the existing literature. This paper designs a non-linear dynamic penalty mechanism to improve the effectiveness of green product quality supervision.

## 3. An evolutionary game model of green product quality supervision

### 3.1 Problem description and basic assumptions

Under the traditional supervision without blockchain, the information about green products has low credibility, and moral issues permeate the entire transaction. Under the supervision with blockchain, due to the unchangeable, transparency and real-time, the program automatically records all process information and logistic information of products, and stores the information on blockchain. Consumers can give a request to the system and receive symmetrical information, and the platform effectively supervises the entire process of green products. In reality, numerous online platforms (e.g., Alibaba, JD.com and Amazon) establishes the traceability system with blockchain, and the manufacturers connect the system to upload all the information including raw materials, process, express and so on. As shown in the Fig 1.

**Fig 1:** Platform blockchain technology operation flowchart.

Consider a supply chain with three players: a product seller, an online platform, and a consumer. They are all bounded rationality players. The seller sells the products through an online platform to the consumer. The format is called agency retailing. The seller’s strategy set is {green products, fake green products, common products}. The online platform’s strategy set is {supervision by blockchain technology, supervision by random inspection}. The consumer’s strategy choice space is {with green consciousness, without green consciousness}. The five crucial assumptions of this model are as follows:

Assumption 1: Online seller chooses to supply green products with the probability of *x*, *x*∈[0,1]. The probability of fake green products among non-green products is *β*, *β*∈[0,1], and the likelihood of common products is (1 − *β*). The online platform chooses to supervise by blockchain technology with the probability of *y*, *y*∈[0,1].Consumer with green consciousness purchase the products with the probability of *z*, *z*∈[0,1].

Assumption 2: The consumer utility of purchasing common goods on the platform is *V*, and the change utility value of consumers with green consciousness purchasing green or non-green goods is *θ*, 0<*θ*<1. Under the agency selling format, the seller sells the products on the online marketplace with a commission fee. When products are sold, the total revenue of selling green products is *M*_*G*_, that of selling common products is *M*_*N*_. *λ* is the proportional fee. For example, JD.com in 2022 charges 6% for books and 3% for fresh food.

Assumption 3: When the online platform chooses to supervise strictly, the cost of using blockchain technology is *C*_*B*_. And if the online platform adopts loose supervision, such as the rate of bad reviews, volume of customer complaints, random inspection of commodities, *etc*., the cost of the random inspection is *C*_*T*_, and *C*_*B*_>*C*_*T*_>0. But if the online platform adopts blockchain technology, consumers’ trust will increase, which will also bring invisible gains to the platform, such as reputation, repurchase, etc. It is denoted by *R*. Under the blockchain technology, the platform finds that the seller provides low-quality products, and it imposes a fine of *F*. Under traditional supervision, the rate of fake green products randomly inspected by platform is *k*.

Assumption 4: Green products refer to products that minimize environmental damage by scientific technology throughout their lifecycle, including package, materials and energy-saving, etc. Compared with ordinary products, green products are made from pollution-free raw materials with 20% to 25% higher cost than ordinary products. The cost of supplying green products for the seller is *C*_*G*_, and the cost of supplying the non-green products is *C*_*N*_, *C*_*G*_>*C*_*N*_>0. Under the blockchain supervision, it is easy to find the product quality on the online platform. The whitewashing cost of fake green products is *C*_*F*_. Once the platform finds the quality problems, the seller must pay the consumer compensation for *C*_*C*_.

Assumption 5: When the consumer purchases fake green products, he (or she) will report to the platform, the cost of the complaint is *C*_*R*_, *C*_*R*_<*C*_*C*_, and the compensation given by the platform to the consumer is *C*_*Q*_, *C*_*R*_<*C*_*C*_ + *C*_*Q*_.

Table 1 includes the parameters and descriptions for the model.

**Table 1:** Parameter.

Symbols	Descriptions
*x*	The probability of online seller supplying green products
*y*	The probability of platform supervising by blockchain technology
*β*	The probability of fake green products among non-green products
*z*	The probability of consumer with green consciousness
*C*_*G*_	The cost of green products
*C*_*N*_	The cost of common products
*C*_*B*_	The cost of strict supervision by blockchain technology
*C*_*T*_	The cost of traditional supervision by random inspection
*F*	Online platform’s penalty cost
*C*_*F*_	The whitewashing cost of fake green products
*C*_*R*_	The cost of consumer complaint
*C*_*Q*_	Consumer’s compensation by platform
*C*_*C*_	Consumer’s compensation by seller
*V*	The common consumer utility of purchasing products
*θ*	The change value of utility of consumer with green conscious
*R*	Invisible gains to the platform
*M*_*G*_	The total revenue of selling green products on online platform
*M*_*N*_	The total revenue of selling common products on online platform
*λ*	The commission rate
*k*	The rate of fake green products randomly inspected by platform

Based on the five assumptions, we get the payoff matrix in Table 2.

**Table 2:** Payoff matrix on online green product quality supervision.

Strategic choice		Consumer	Seller		
			Green products *x*	Non-green products 1 − *x*	
				Fake green product *β*	Common product 1 − *β*
**Online platform**	Supervision by blockchain technology *y*	Green consciousness *z*	(1 − *λ*) *M*_*G*_ − *C*_*G*_; *λM*_*G*_ + *R* − *C*_*B*_; (1 + *θ*)*V* − *M*_*G*_	(1 − *λ*) *M*_*G*_ − *C*_*N*_ − *C*_*F*_ − *F* − *C*_*C*_;*λM*_*G*_ − *C*_*B*_ + *F* − *C*_*Q*_;(1 − *θ*)*V* − *M*_*G*_ − *C*_*R*_ + *C*_*C*_ + *C*_*Q*_	(1 − *λ*) *M*_*N*_ − *C*_*N*_; *λM*_*N*_ − *C*_*B*_; (1 − *θ*)*V* − *M*_*N*_
		No green consciousness 1 − *z*	(1 − *λ*) *M*_*G*_ − *C*_*G*_; *λM*_*G*_ + *R* − *C*_*B*_; *V* − *M*_*G*_	(1 − *λ*) *M*_*G*_ − *C*_*N*_ − *C*_*F*_ − *F*;*λM*_*G*_ − *C*_*B*_ + *F*; *V* − *M*_*G*_	(1 − *λ*) *M*_*N*_ − *C*_*N*_; *λM*_*N*_ − *C*_*B*_; *V* − *M*_*N*_
	Supervision by random inspection 1 − *y*	Green consciousness *z*	(1 − *λ*) *M*_*G*_ − *C*_*G*_; *λM*_*G*_ − *C*_*T*_; (1 + *θ*)*V* − *M*_*G*_	(1 − *λ*) *M*_*G*_ − *C*_*N*_ − *C*_*F*_ − *kF* − *C*_*C*_;*λM*_*G*_ − *C*_*T*_ + *kF* − *C*_*Q*_;(1 − *θ*)*V* + *C*_*C*_ + *C*_*Q*_ − *C*_*R*_ − *M*_*G*_	(1 − *λ*) *M*_*N*_ − *C*_*N*_; *λM*_*N*_ − *C*_*T*_; (1 − *θ*)*V* − *M*_*N*_
		No green consciousness 1 − *z*	(1 − *λ*) *M*_*G*_ − *C*_*G*_; *λM*_*G*_ − *C*_*T*_; *V* − *M*_*G*_	(1* − λ*) *M*_*G*_ − *C*_*N*_ − *C*_*F*_ − *kF*;*λM*_*G*_ − *C*_*T*_ + *kF*;*V* − *M*_*G*_	(1 − *λ*) *M*_*N*_ − *C*_*N*_; *λM*_*N*_ − *C*_*T*_; *V* − *M*_*N*_

### 3.2 The game analysis under the static penalty mechanism

(1) Based on the above payoff matrix for online green product quality supervision, the expected revenue of seller choosing to supply green product is

$$\begin{array}{c} E_{A}=yz\left[(1-\lambda )M-C_{G}\right]+z(1-y)\left[(1-\lambda )M-C_{G}\right]+y(1-z)[(1-\lambda )M-\left.C_{G}\right]\\ +(1-y)(1-z)\left[(1-\lambda )M-C_{G}\right]=(1-\lambda )M_{G}-C_{G} \end{array}$$ (1)

The expected revenue of the seller choosing to supply fake green and common product is

$$\begin{array}{l} E_{A1}=yz\left\{\beta \left[(1-\lambda )M_{G}-C_{N}-C_{F}-F-C_{C}\right]+(1-\beta )\left[(1-\lambda )M_{N}-C_{N}\right]\right\}+(1-\text{y})z\left\{\beta \left[(1-\lambda )M_{G}-C_{N}-C_{F}-kF-C_{C}\right]+(1-\beta )\left[(1-\lambda )M_{N}-C_{N}\right]\right\}\\ +y(1-z)\{\beta [(1-\lambda )\left.\left.M_{G}-C_{N}-C_{F}-F\right]+(1-\beta )\left[(1-\lambda )M_{N}-C_{N}\right]\right\}+(1-y)(1-z)\left\{\beta \left[(1-\lambda )M_{G}-\left.C_{N}-C_{F}-kF\right]\right.\left.+(1-\beta )\left[(1-\lambda )M_{N}-C_{N}\right]\right\}\right. \end{array}$$ (2)

The average expected revenue can be calculated as

$$\bar{E_{A}}=xE_{A}+(1-x)E_{A1}$$ (3)

The consequent replicator dynamics equation of *x* is:

$$\begin{array}{l} F(x)=dx/dt=x\left(E_{A}-\bar{E_{A}}\right)=x(1-x)\left\{\left(1-\lambda )\left(M_{G}-M_{N}\right)-C_{G}+C_{N}-\beta [(1-\lambda \right)\right.\\ \left.\left.M_{G}-C_{N}-C_{F}-yF-(1-y)kF-zC_{C}\right]\right\} \end{array}$$ (4)

The derivative of the replicator dynamics equation of *x* can be further calculated below:

$$\begin{array}{l} dF(x)/dx=(1-2x)\left\{(1-\lambda )\left(M_{G}-M_{N}\right)-C_{G}+C_{N}-\beta \left[(1-\lambda )M_{G}-C_{N}-C_{F}-\right.\right.\\ \left.\left.yF-(1-y)kF-zC_{C}\right]\right\} \end{array}$$ (5)

The function on *y* can be set to *G*(*y*), giving:

$$\begin{array}{l} G(y)=(1-\lambda )\left(M_{G}-M_{N}\right)-C_{G}+C_{N}-\beta \left[(1-\lambda )M_{G}-C_{N}-C_{F}-yF-(1-\right.\\ \text{y})kF-zC_{C}] \end{array}$$ (6)

According to the stability theorem of the differential equation, the likelihood of the seller supplying green product in a stable state must be satisfied: *F*(*x*) = 0 and *dF*(*x*)⁄*dx*<0. Since *∂G*(*y*)⁄*∂y*>0, when $y=y^{*},G(y)=0,dF(y)/dy\equiv 0$ and the seller cannot have a certain strategy; when *$y>y^{*},G(y)>0,dF(x)/dx|x=1<0$* and *x* = 1 is ESS; conversely, *x* = 0 is ESS. Therefore, With the increase of the probability of supervision by blockchain technology, the seller’s stable strategy will be shifted to sell green products. When the probability decreases, the seller is inclined to sell non-green products.

(2) The expected revenue of platform supervising by blockchain technology is

$$\begin{array}{l} E_{B}=xz\left(\lambda M_{G}+R-C_{B}\right)+z(1-x)\left[\beta \left(\lambda M_{G}-C_{B}+F-C_{Q}\right)+(1-\beta )\left(\lambda M_{N}-\left.\left.C_{B}\right)\right]\right.\right.\\ +x(1-z)\left(\lambda M_{G}+R-C_{B}\right)+(1-x)(1-z)\left[\beta \left(\lambda M_{G}-C_{B}+F\right)+(1-\beta )\left(\lambda M_{N}-\right.\right.C_{B})] \end{array}$$ (7)

The expected revenue of platform supervising by random inspection is

$$\begin{array}{l} E_{B1}=xz\left(\lambda M_{G}-C_{T}\right)+(1-x)z\left[\beta \left(\lambda M_{G}-C_{T}+kF-C_{Q}\right)+(1-\beta )\left(\lambda M_{N}-C_{T}\right)\right]+\\ x(1-z)\left(\lambda M_{G}-C_{T}\right)+(1-x)(1-z)\left[\beta \left(\lambda M_{G}-C_{T}+kF\right)+(1-\beta )\left(\lambda M_{N}-C_{T}\right)\right] \end{array}$$ (8)

The average expected revenue can be worked out as

$$\bar{E_{B}}=yE_{B}+(1-y)E_{B1}$$ (9)

The replicator dynamic equation about the platform can be further worked out below:

$$F(y)=dy/dt=y(1-y)\left[xR-C_{B}+C_{T}+\beta (1-x)(1-k)F\right]$$ (10)

The derivative of the replicator dynamics equation of *y* can be determined as

$$dF(y)/dy=(1-2y)\left[xR-C_{B}+C_{T}+\beta (1-x)(1-k)F\right]$$ (11)

The function on *x* can be set to *H*(*x*), giving:

$$H(x)=xR-C_{B}+C_{T}+\beta (1-x)(1-k)F$$ (12)

According to the stability theorem of the differential equation, the likelihood of the platform choosing to supervise by blockchain technology in a stable state must be satisfied: *F*(*y*) = 0 and *dF*(*y*)⁄*dy*<0. Since *∂H*(*x*)⁄*∂x*<0,when $x=x^{*},H(x)=0,dF(y)/dy\equiv 0$ and the platform cannot have a certain strategy; when $x<x^{*},H(x)>0,dF(y)/dy|y=1<0$ and *y* = 1 is ESS; conversely, *y* = 0 is ESS. Therefore, With the increased probability of selling non-green products, the platform’s stable strategy will be shifted to supervise by blockchain technology. When the probability decreases, the platform is inclined to supervise by random inspection.

(3) The expected revenue of the consumer with green consciousness is

$$\begin{array}{l} E_{C}=xy\left[(1+\theta )V-M_{G}\right]+x(1-y)\left[(1+\theta )V-M_{G}\right]+y(1-x)\left.\left.\{\beta [(1-\theta )V-M_{G}-C_{R}+C_{C}+C_{Q}\right]+(1-\beta )\left[(1-\theta )V-M_{N}\right]\right\}\\ +(1-x)(1-y)\left.\left.\left\{\beta \left[(1-\theta )V-M_{G}\right.\right.-C_{R}+C_{C}+C_{Q}\right]+(1-\beta )\left[(1-\theta )V-M_{N}\right]\right\} \end{array}$$ (13)

The expected revenue of the consumer without green consciousness is

$$\begin{array}{l} E_{C1}=xy\left(\text{V}-M_{G}\right)+(1-x)y\left[\beta \left(\text{V}-M_{G}\right)+(1-\beta )\left(\text{V}-M_{N}\right)\right]+x(1-y)(\text{V}-\left.M_{G}\right)\\ +(1-x)(1-y)\left[\beta \left(\text{V}-M_{G}\right)+(1-\beta )\left(\text{V}-M_{N}\right)\right] \end{array}$$ (14)

The average expected revenue can be calculated as

$$\bar{E_{c}}=zE_{c}+(1-z)E_{C1}$$ (15)

The replicator dynamic equation of the consumer can be further calculated below:

$$F(z)=dz/dt=z(1-z)\left[(2x-1)\theta V+(1-x)\beta \left(C_{C}+C_{Q}-C_{R}\right)\right]$$ (16)

The derivative of the replicator dynamics equation of *z* can be determined as

$$dF(z)/dz=(1-2z)\left[(2x-1)\theta V+(1-x)\beta \left(C_{C}+C_{Q}-C_{R}\right)\right]$$ (17)

The function on *x* can be set to *J*(*x*), giving:

$$J(x)=(2x-1)\theta V+(1-x)\beta \left(C_{C}+C_{Q}-C_{R}\right)$$ (18)

According to the stability theorem of the differential equation, the probability of the consumer selling high-quality products in a stable state must be satisfied: *F*(*z*) = 0 and *dF*(*z*)⁄*dz*<0. Since *∂J*(*x*)⁄*∂x*>0, when $x=x^{**},J(x)=0,dF(z)/dz\equiv 0$ and the seller cannot have a certain strategy; when *$x<x^{**},J(x)<0,dF(z)/dz|z=0<0$* and *z* = 0 is ESS; conversely, *z* = 1 is ESS. Therefore, with the increase of the probability of selling green products, the consumer improves the green consciousness. When the probability decreases, the consumer will keep the non-green consciousness.

(4) Stability analysis of strategy combination

According to the Lyapunov’s First Method, if the Jacobi matrix eigenvalues are negative, the equilibrium solution is an evolutionary stable strategy (ESS); conversely, the equilibrium solution is an unstable strategy. This paper discusses the stability of pure strategy equilibrium solutions. We can obtain the following matrix on the basis of replicator dynamic equations.


$$J=\left[\begin{array}{c} \frac{\partial F(x)}{\partial x}\;\;\frac{\partial F(x)}{\partial y}\;\;\frac{\partial F(x)}{\partial z}\\ \frac{\partial F(y)}{\partial x}\;\;\frac{\partial F(y)}{\partial y}\;\;\frac{\partial F(y)}{\partial z}\\ \frac{\partial F(z)}{\partial x}\;\;\;\frac{\partial F(z)}{\partial y}\;\;\frac{\partial F(z)}{\partial z} \end{array}\right]=\left[\begin{array}{c} a_{11\;\;}a_{12}\;\;a_{13}\\ a_{21}\;\;a_{22}\;\;a_{23}\\ a_{31}\;\;a_{32}\;\;a_{33} \end{array}\right]$$ (19)

$$a_{11}=\left\{(1-\lambda )\left(M_{G}-M_{N}\right)-C_{G}+C_{N}-\beta \left[(1-\lambda )M_{G}-C_{N}-C_{F}-yF-(1-y)kF-\right.\right.zC_{c}]\}$$ (20)

$$a_{12}=x(1-x)(1-k)\beta F$$ (21)

$$a_{13}=x(1-x)\beta C_{C}$$ (22)

$$a_{21}=y(1-y)[R-\beta (1-k)F]$$ (23)

$$a_{22}=(1-2y)\left[xR-C_{B}+C_{T}+\beta (1-x)(1-k)F\right]$$ (24)

$$a_{23}=0$$ (25)

$$a_{31}=z(1-z)\left[2\theta V-\beta \left(C_{R}-C_{C}-C_{Q}\right)\right]$$ (26)

$$a_{32}=0$$ (27)

$$a_{33}=(1-2z)\left[(2x-1)\theta V+(1-x)\beta \left(C_{C}+C_{Q}-C_{R}\right)\right]$$ (28)

Table 3 presents the analytical results of the equilibrium points.

**Table 3:** Stability analysis under static penalty mechanism.

Equilibrium point	Eigenvalues *λ*_1_	Eigenvalues *λ*_2_	Eigenvalues *λ*_3_
(0,0,0)	*C*_*T*_ − *C*_*B*_ + *βF*	*β*(*C*_*C*_ − *C*_*R*_ + *C*_*Q*_) − *θV*	*C*_*N*_ − *C*_*G*_ + (1 − *λ*)(*M*_*G*_ − *M*_*N*_) − (1 − *λ*)*βM*_*G*_ + *β*(*kF* + *C*_*F*_ + *C*_*N*_)
(1,0,0)	*θV*	*C*_*T*_ − *C*_*B*_ + *R*	*C*_*G*_ − *C*_*N*_ − (1 − *λ*)(*M*_*G*_ − *M*_*N*_) + (1 − *λ*)*βM*_*G*_ − *β*(*kF* + *C*_*F*_ + *C*_*N*_)
(0,1,0)	*C*_*B*_ − *C*_*T*_ − *βF*	*β*(*C*_*C*_ − *C*_*R*_ + *C*_*Q*_) − *θV*	*C*_*N*_ − *C*_*G*_ + (1 − *λ*)(*M*_*G*_ − *M*_*N*_) − (1 − *λ*)*βM*_*G*_ + *β*(*F* + *C*_*F*_ + *C*_*N*_)
(0,0,1)	*C*_*T*_ − *C*_*B*_	*β*(*C*_*R*_ − *C*_*C*_ + *C*_*Q*_) + *θV*	*C*_*N*_ − *C*_*G*_ + (1 − *λ*)(*M*_*G*_ − *M*_*N*_) − (1 − *λ*)*βM*_*G*_ + *β*(*kF* + *C*_*F*_ + *C*_*N*_ + *C*_*C*_)
(1,1,0)	*θV*	*C*_*B*_ − *C*_*T*_ − *R*	*C*_*G*_ − *C*_*N*_ − (1 − *λ*)(*M*_*G*_ − *M*_*N*_) + (1 − *λ*)*βM*_*G*_ − *β*(*F* + *C*_*F*_ + *C*_*N*_)
(1,0,1)	* − θV*	*C*_*T*_ − *C*_*B*_ + *R*	*C*_*G*_ − *C*_*N*_ − (1 − *λ*)(*M*_*G*_ − *M*_*N*_) + (1 − *λ*)*βM*_*G*_ − *β*(*kF* + *C*_*F*_ + *C*_*N*_ + *C*_*C*_)
(0,1,1)	*C*_*B*_ − *C*_*T*_	*β*(*C*_*R*_ − *C*_*C*_ + *C*_*Q*_) + *θV*	*C*_*N*_ − *C*_*G*_ + (1 − *λ*)(*M*_*G*_ − *M*_*N*_) − (1 − *λ*)*βM*_*G*_ + *β*(*F* + *C*_*F*_ + *C*_*N*_ + *C*_*C*_)
(1,1,1)	* − θV*	*C*_*B*_ − *C*_*T*_ − *R*	*C*_*G*_ − *C*_*N*_ − (1 − *λ*)(*M*_*G*_ − *M*_*N*_) + (1 − *λ*)*βM*_*G*_ − *β*(*F* + *C*_*F*_ + *C*_*N*_ + *C*_*C*_)

The following scenarios can be seen in Table 4.

**Table 4:** Stability analysis of different scenarios under static penalty mechanism.

Equilibrium point	*β*(*C*_*C*_ + *C*_*Q*_ − *C*_*R*_)<*θV*		*θV*<*β*(*C*_*C*_ + *C*_*Q*_ − *C*_*R*_)<2*θV*			
	Scenario 1	Stability	Scenario 2	Stability	Scenario 3	Stability
(0,0,0)	( + , + ,-)	Unstable	( + , + ,-)	Unstable	( + , + ,-)	Unstable
(1,0,0)	( + , + ,-)	Unstable	( + , + ,-)	Unstable	( + , + ,-)	Unstable
(0,1,0)	(-,-, + )	Unstable	(-, + , + )	Unstable	(-, + , + )	Unstable
(0,0,1)	(-, + ,±)	Unstable	(-,-, + )	Unstable	(-,-,-)	ESS
(1,1,0)	( + ,-,-)	Unstable	( + ,-,-)	Unstable	( + ,-, + )	Unstable
(1,0,1)	(-, + ,-)	Unstable	(-, + , + )	Unstable	(-, + , + )	Unstable
(0,1,1)	( + , + , + )	Unstable	( + ,- , + )	Unstable	( + ,- , + )	Unstable
(1,1,1)	(-,-,-)	ESS	(-,-,-)	ESS	(-,-,-)	ESS

**Scenario 1:** if condition *β*(*C*_*C*_ + *C*_*Q*_ − *C*_*R*_)<*θV* is satisfied, it shows when green conscious consumers buy fake green products, the compensations they received are difficulty to make up for the reduced effectiveness of buying fake products, (1,1,1) becomes evolutionary stable strategy combinations.

**Scenario 2:** if condition $\theta V<\beta \left(C_{C}+C_{Q}-C_{R}\right)<2\theta V,C_{G}-C_{N}-(1-\lambda )\left(M_{G}-\right.\left.M_{N}\right)+(1-\lambda )\beta M_{G}<\beta \left(kF+C_{F}+C_{N}+C_{C}\right)$ are satisfied, it shows when the compensations can make up for the green conscious consumer’s reduced effectiveness of buying fake products, and the cost saved by non-green products cannot cover whitewashing cost, consumer compensation and penalties, (1,1,1) may become evolutionary stable strategy combinations.

**Scenario 3:** if conditions $\theta V<\beta \left(C_{C}+C_{Q}-C_{R}\right)<2\theta V,\beta \left(kF+C_{F}+C_{N}+C_{C}\right)<C_{G}-C_{N}-(1-\lambda )\left(M_{G}-M_{N}\right)+(1-\lambda )\beta M_{G}<\beta \left(F+C_{F}+C_{N}+C_{C}\right)$ are satisfied, it indicates that the compensations can make up for the green conscious consumer’s reduced effectiveness of buying green fake products, and the cost saved by non-green products cannot cover whitewashing cost, consumer compensation and penalties, (1,1,1),(0,0,1) become stable strategy combinations.

Under the static penalty mechanism, the compensation and the cost saved by non-green products are the decisive factors of the best evolutionary stable strategy combination. This shows that the improvement of consumers’ green awareness has driven sellers to sell green products to some extent, and makes the platform attach more importance to strengthening the supervision of fake green products by blockchain technology.

### 3.3 The game analysis under the dynamic penalty mechanism

Assuming that the penalties are related to the probability of selling non-green products, it means that the higher probability that a seller sells non-green products, the less penalties; conversely, the greater penalties.

Setting the fixed penalties into linear function $F(x)=-f_{m}x^{2}+f_{m},f_{m}$ is the highest penalties. The formula indicates that when sellers sell green products (*x* = 1), the platform will not impose any penalties on the sellers; When sellers sell non-green products (*x*∈[0,1)), the platform will impose penalties based on the degree of selling non-green products by sellers.

Therefore, the consequent replicator dynamics equations of online platform, consumer and seller become:

$$F_{1}(x)=x(1-x)\left\{(1-\lambda )\left(M_{G}-M_{N}\right)-C_{G}+C_{N}-\beta \left[(1-\lambda )M_{G}-C_{N}-C_{F}-y(1-\right.\right.\left.\left.\left.x^{2}\right)f_{m}-(1-y)k\left(1-x^{2}\right)f_{m}-zC_{C}\right]\right\}$$ (29)

$$F_{1}(y)=y(1-y)\left[xR-C_{B}+C_{T}+\beta (1-x)(1-k)\left(1-x^{2}\right)f_{m}\right]$$ (30)

$$F_{1}(z)=z(1-z)\left[(2x-1)\theta V+(1-x)\beta \left(C_{C}+C_{Q}-C_{R}\right)\right]$$ (31)

According to the replicator dynamic equations, we can obtain the following Jacobi matrix.


$$J=\left[\begin{array}{c} b_{11}\;\;b_{12}\;\;b_{13}\\ b_{21}\;\;b_{22}\;\;b_{23}\\ b_{31}\;\;b_{32}\;\;b_{33} \end{array}\right]$$ (32)

$$b_{11}=(1-2x)\left\{(1-\lambda )\left(M_{G}-M_{N}\right)-C_{G}+C_{N}-\beta \left[(1-\lambda )M_{G}-C_{N}-C_{F}-zC_{C}\right]\right\}+\beta \left(1-3x^{2}-2x+4x^{3}\right)f_{m}[(1-k)y+k]$$ (33)

$$b_{12}=x(1-x)\left(1-x^{2}\right)(1-k)f_{m}$$ (34)

$$b_{13}=x(1-x)\beta C_{C}$$ (35)

$$b_{21}=y(1-y)\left[R-\beta (1-k)\left(1-3x^{2}f_{m}\right)\right]$$ (36)

$$b_{22}=(1-2y)\left[xR-C_{B}+C_{T}+\beta (1-x)(1-k)\left(1-x^{2}\right)f_{m}\right]$$ (37)

$$b_{23}=0$$ (38)

$$a_{31}=z(1-z)\left[2\theta V-\beta \left(C_{R}-C_{C}-C_{Q}\right)\right]$$ (39)

$$a_{32}=0$$ (40)

$$a_{33}=(1-2z)\left[(2x-1)\theta V+(1-x)\beta \left(C_{C}+C_{Q}-C_{R}\right)\right]$$ (41)

**Scenario 4:** under the dynamic penalty mechanism, if conditions $C_{G}-C_{N}-(1-\lambda )\left(M_{G}-M_{N}\right)+(1-\lambda )\beta M_{G}<\beta \left(C_{F}+C_{N}+C_{C}\right)$ are satisfied, showing that the cost saved by selling non-green products is hard to pay for whitewashing fees and consumer compensation costs, (1,1,1) become the only optimal stable strategy combination, as shown in Table 5.

**Table 5:** Stability analysis under dynamic penalty mechanism.

Equilibrium point	Eigenvalues				Stability
	*λ*_1_	*λ*_2_	*λ*_3_	Sign	
(0,0,0)	*β*(*C*_*C*_ − *C*_*R*_ + *C*_*Q*_) − *θV*	*C*_*T*_ − *C*_*B*_ + (1 − *k*)*βR*	*C*_*N*_ − *C*_*G*_ + (1 − *λ*)(*M*_*G*_ − *M*_*N*_) − (1 − *λ*)*βM*_*G*_ + *β*(*kF* + *C*_*F*_ + *C*_*N*_)	(±, −, + )	Unstable
(1,0,0)	*θV*	*C*_*T*_ − *C*_*B*_ + *R*	*C*_*G*_ − *C*_*N*_ − (1 − *λ*)(*M*_*G*_ − *M*_*N*_) + (1 − *λ*)*βM*_*G*_ − *β*(*C*_*F*_ + *C*_*N*_)*	( + , + , −)	Unstable
(0,1,0)	*C*_*B*_ − *C*_*T*_ − *βF*	*C*_*B*_ − *C*_*T*_ − (1 − *k*)*βR*	*C*_*N*_ − *C*_*G*_ + (1 − *λ*)(*M*_*G*_ − *M*_*N*_) − (1 − *λ*)*βM*_*G*_ + *β*(*F* + *C*_*F*_ + *C*_*N*_)	(±, −, + )	Unstable
(0,0,1)	*β*(*C*_*C*_ − *C*_*R*_ + *C*_*Q*_) − *θV*	*C*_*T*_ − *C*_*B*_ + (1 − *k*)*βR*	*C*_*N*_ − *C*_*G*_ + (1 − *λ*)(*M*_*G*_ − *M*_*N*_) − (1 − *λ*)*βM*_*G*_ + *βC*_*F*_ + *C*_*N*_ + *C*_*C*_)	(±, −, + )	Unstable
(1,1,0)	*θV*	*C*_*B*_ − *C*_*T*_ − *R*	*C*_*G*_ − *C*_*N*_ − (1 − *λ*)(*M*_*G*_ − *M*_*N*_) + (1 − *λ*)*βM*_*G*_ − *β*(*C*_*F*_ + *C*_*N*_)	( + , −, + )	Unstable
(1,0,1)	* − θV*	*C*_*T*_ − *C*_*B*_ + *R*	*C*_*G*_ − *C*_*N*_ − (1 − *λ*)(*M*_*G*_ − *M*_*N*_) + (1 − *λ*)*βM*_*G*_ − *β*(*C*_*F*_ + *C*_*N*_ + *C*_*C*_)	(−, + , −)	Unstable
(0,1,1)	*β*(*C*_*R*_ − *C*_*C*_ − *C*_*Q*_) + *θV*	*C*_*B*_ − *C*_*T*_ − (1 − *k*)*βR*	*C*_*N*_ − *C*_*G*_ + (1 − *λ*)(*M*_*G*_ − *M*_*N*_) − (1 − *λ*)*βM*_*G*_ + *β*(*F* + *C*_*F*_ + *C*_*N*_ + *C*_*C*_)	(±, −, + )	Unstable
(1,1,1)	* − θV*	*C*_*B*_ − *C*_*T*_ − *R*	*C*_*G*_ − *C*_*N*_ − (1 − *λ*)(*M*_*G*_ − *M*_*N*_) + (1 − *λ*)*βM*_*G*_ − *β*(*C*_*F*_ + *C*_*N*_ + *C*_*C*_)	(−, −, −)	ESS

*$C_{G}-C_{N}-(1-\lambda )\left(M_{G}-M_{N}\right)+(1-\lambda )\beta M_{G}<\beta \left(C_{F}+C_{N}+C_{C}\right)$

Under the dynamic punishment mechanism, the platform implements the blockchain supervision technology, when the cost saved by non-green products cannot cover the cost of whitewashing and consumer compensation, the green products become the best strategic choice for sellers. The dynamic penalty mechanism reduces the possibility of (0,0,1) becoming a stable strategy combination.

## 4. Numerical simulation analysis

To confirm the validity of the conclusions, and straightforwardly show the impact of each parameter changed on the game, this study performs numerical evolution and simulation analysis by MATLAB 2020b to simulate the game process.

### 4.1 Simulation of the evolution of each party’s strategic choices

Under the static penalty mechanism, the values of the factors are as follows: $M_{G}=150,M_{N}=100,C_{B}=100,C_{G}=90,C_{T}=80,F=60,C_{F}=40,C_{C}=40,R=30,C_{R}=10,C_{Q}=20,V=80,\theta =0.3,\beta =0.3,k=0.3,\lambda =0.1.$ The factors satisfy the condition that *β*(*C*_*C*_ + *C*_*Q*_ − *C*_*R*_)<*θV*, and evolve over 50 times from different initial strategy combinations. The results can be illustrated in Fig 2.

**Fig 2:** Simulation diagram of scenario 1.

Setting these values that *V* = 40, *F* = 100 to satisfy *θV* < *β*(*C*_*C*_ + *C*_*Q*_ − *C*_*R*_)<2*θV*, and $C_{G}-C_{N}-(1-\lambda )\left(M_{G}-M_{N}\right)+(1-\lambda )\beta M_{G}<\beta \left(kF+C_{F}+C_{N}+C_{C}\right)$, and evolve over 50 times from different initial strategy combinations. Therefore, there are one stable point, and the simulation results are presented in Fig 3.

**Fig 3:** Simulation diagram of scenario 2.

We adjust *V* = 40, *F* = 60 to satisfy the condition *θV* < *β*(*C*_*C*_ + *C*_*Q*_ − *C*_*R*_)<2*θV* and $\beta \left(kF+C_{F}+\right.\left.C_{N}+C_{C}\right)<C_{G}-C_{N}-(1-\lambda )\left(M_{G}-M_{N}\right)+(1-\lambda )\beta M_{G}<\beta \left(F+C_{F}+C_{N}+C_{C}\right),$ there exists the only optimal stable point, and its simulation results are shown in Fig 4.

**Fig 4:** Simulation diagram of scenario 3.

Under the dynamic penalty mechanism, the values of the factors are as follows: $M_{G}=150,M_{N}=100,C_{B}=100,C_{G}=90,C_{T}=80,F=150,C_{F}=100,C_{C}=40,R=30,C_{R}=10,C_{Q}=20,V=80,\theta =0.3,\beta =0.3,k=0.3,\lambda =0.1.$ The previous initial parameter settings satisfy the following conditions: $C_{G}-C_{N}-(1-\lambda )\left(M_{G}-M_{N}\right)+(1-\lambda )\beta M_{G}<\beta \left(C_{F}+C_{N}+C_{C}\right)$, and evolve over 50 times from different initial strategy combinations. The simulation is presented in Fig 5.

**Fig 5:** Simulation diagram of scenario 4.

### 4.2 Comparative analysis of seller’s choice evolution under different penalty mechanisms

Under two penalty mechanisms, the values of parameters are the same with the previous parameters and the four initial states of (*x*, *y*, *z*) are simulated with different probabilities (0.2,0.2,0.2),(0.3,0.3,0.3),(0.5,0.5,0.5),(0.7,0.7,0.7), to analyze the impact of different penalty mechanisms to seller’s choice evolution.

As shown in Fig 6, under the dynamic and static punishment mechanism, the probability of selling high-quality products gradually converges and stabilizes after a short shock. Under the dynamic penalty mechanism, when the platform is confronted with quality problems, with the increase of the evolution times, the evolution speed and effect of selling green products are better than those under the static penalty mechanism. However, if there are fewer quality problems on the platform, the impact of the two punishment mechanisms on regulating the fake green products is not obvious. Therefore, when the platform market is filled with fake green products, the dynamic penalty mechanism is more effective and rapid for improving the platform’s market environment and the quality of green products. An effective penalty mechanism will promote the order and stability of the market and protect the rights and interests of consumers.

**Fig 6:** Comparison chart of seller’s strategy evolution under different penalty mechanisms. (a) initial probabilities of all parties is(**0.2,0.2,0.2**). (b) initial probabilities of all parties is(0.3,0.3,0.3). (c) initial probabilities of all parties is(0.4,0.4,0.4). (d) initial probabilities of all parties is(0.5,0.5,0.5).

### 4.3 Comparative analysis of seller’s choice evolution under different supervision technologies

The parameters are set as before, and the four initial states of are simulated with different probabilities (0.2/0.3,0.1,0.5),(0.2/0.3,0.2,0.5),(0.2/0.3,0.5,0.5),(0.2/0.3,0.9,0.5), to analyze the impact of seller’s choice evolution under different supervision technologies. The evolution results are shown in Fig 7.

**Fig 7:** Comparison chart of seller’s choice evolution under different supervision technologies. (a) and (c) are the static punishment mechanism. (b) and (d) are the dynamic punishment mechanism.

Under the static punishment mechanism, Fig 6 shows that when the green conscious consumers are certain, sellers tend to sell non-green products, and the platform adopts random inspection supervision, the final behavior strategy of seller will be further promoted to sell non-green products; Under the two kinds of punishment mechanisms, when the probability of blockchain supervision adopted by the platform increases, the probability of the seller’s choice to sell green products further tends to be 1. In addition, under the same conditions, the dynamic punishment mechanism makes the evolution speed and effect of green products sold by sellers superior to the static punishment mechanism. Therefore, when the platform puts the static penalty mechanism and random inspection supervision into practice, sellers will choose to sell non-green products, and the platform’s quality problems will be more than those under blockchain supervision. Blockchain technology plays a vital role in the supervision of the platform’s fake products. Meanwhile, the dynamic punishment mechanism can speed up the management of sellers’ sales of fake green products.

## 5. Conclusions and suggestions

This paper constructs an evolutionary game model and introduces the dynamic and static punishment mechanisms for green product quality supervision. Based on Lyapunov’s First Method, we discuss the conditions for the existence of the evolutionary stability point. After simulation with MATLAB2020b, the effects of different punishment mechanisms on the evolutionary equilibrium are compared.

The main results are as follows. Firstly, under the static punishment mechanism, the level of the consumers’ green awareness, the compensation for green consumers, and the cost saved by non-green products are the key factors to determine the system evolution. Under the dynamic punishment mechanism, it is essential for the platform to ensure high quality of green products that whether the cost saved by the non-green products can pay whitewashing costs and consumer compensation. The cost of green products is higher than that of common products 20%~25% [39], and the price of green products is generally higher than that of common products, so the excess profit is the fundamental reason to sell fake green products.

Secondly, the combine effect of dynamic punishment and blockchain supervision can effectively and rapidly improve the quality of green products. When the platform adopts random inspection supervision, sellers tend to sell fake green products. It leads to the frequent occurrence of the green product quality problems. When the platform implements blockchain supervision, the dynamic punishment mechanism is obviously superior to the static punishment mechanism, regardless of the evolution speed or the evolution effect. The traceability and integrity of the blockchain help the platform to improve asymmetry information, while the dynamic punishment mechanism further increases the penalty and risk of fake green products supplied by sellers.

Thirdly, the improvement of consumers’ green awareness can drive sellers to sell green products, and make the platform strengthen the supervision of fake green products. Under the static punishment mechanism, when consumers’ green awareness has been improved, and they purchase fake green products, this increases their disappointment. Meanwhile, if this disappointment is far greater than the compensation from the platform and the seller, the likelihood of consumer’s complaint will increase. Then, in order to achieve a stable system, the probability of selling green products and blockchain supervision also increase. Therefore, the green awareness of consumers is an essential factor to promote the quality of green products.

The findings of this study offer suggestions for the parties. For the platform, when confronted with the dilemma of fake green products, they can apply blockchain technology or set up dynamic punishment mechanism to increase the difficulty and cost of counterfeiting. The joint effect can speed up the management of fake green products and improve the quality of the platform’s green products. For the government, they can give the support to the platform for the applied of blockchain. Financial support or tax reduction can encourage enterprises to supervise green product quality and reduce their burden to promote sustainable development. Governments play a vital role as a moderating in predicting green product buying attitudes [40]. Under the "Carbon Peaking and Carbon Neutrality", China Sustainable Consumption Research Program in 2023 announced that nearly half of the interviewees have consciously consumed green products in the past year.

## 6. Limitation and future research

This study considers the platform, sellers and consumers, but the role of government departments is also hard to ignore. In future research, government departments can be involved in the evolutionary game to be discussed. Future research can further overcome the difficulty of simulation data and make the findings more applicable to the platform management.
